The article "The Function of circRNA-0047604 in Regulating the Tumor Suppressor Gene DACH1 in Breast Cancer" was retracted in 2024. Reasons: signs of a paper mill; suspected computer-generated content; unreliable results or conclusions; concerns about the data.

# The Function of circRNA-0047604 in Regulating the Tumor Suppressor Gene DACH1 in Breast Cancer

**DOI:** 10.1155/2022/6589651

**Published:** 2022-01-20

**Authors:** Bingkun Zhao, Rong Zhou, Changle Ji, Diya Liu, Tianqi Wu, Hui Xu, Dongmei Lan, Chao Yao, Yuanzhi Xu, Lin Fang

**Affiliations:** ^1^Department of Stomatology, Shanghai Tenth People's Hospital, Tongji University School of Medicine, Shanghai 200072, China; ^2^Department of Breast and Thyroid Surgery, Shanghai Tenth People's Hospital, Shanghai 200072, China; ^3^Department of Plastic Surgery, Affiliated Hospital of Xuzhou Medical University, Xuzhou, Jiangsu 221000, China; ^4^Medical College of Anhui University of Science and Technology, Huainan, Anhui 232000, China

## Abstract

Breast cancer is the most common cancer among females. Dachshund Homolog 1 (DACH1) gene is regarded as an important tumor suppressor gene in breast cancer which plays an important regulatory role in the development disease progression, particularly in carcinomas. Circular RNAs (circRNAs) and microRNA (miRNA), regarded as a novel group of noncoding RNAs, are always involved in regulating gene expression. In this work, hsa_circ_0047604 expressed lower in breast cancer tissue and played the role of sponge of miR-548o. By this way, hsa_circ_0047604 could upregulate DACH1 to inhibit breast cancer. In conclusion, this study revealed that hsa_circ_0047604 acted as a tumor suppressor and regulated breast cancer progression via hsa_circ_0047604–miR-548o–DACH1 axis, which might provide a therapeutic method for breast cancer.

## 1. Introduction

Breast cancer is one of the most common cancers, accounting for 23% of female malignant tumors. It is the second leading cause of cancer-related death in women worldwide [1]. Although great progress has been made in recent years to improve the development of an earlier diagnosis, tumor recurrence and distant metastasis remain the most pressing problem to be solved.

Dachshund Homolog 1 (DACH1) is a member of the DACH family and plays an essential role in promoting the differentiation of the *Drosophila* eye and limb subfamily of nuclear protein [2]. Results from a recent study of more than 2,000 human breast cancer cases indicate that reduction of DACH1 is correlated with a poor breast cancer prognosis [3]. Accordingly, it is found that it can inhibit breast tumor growth and suppress oncogene-induced breast cancer cell migration and invasion [3, 4]. Moreover, DACH1 is involved in a broad variety of signal transduction pathways and may act as a significant target gene for ER (estrogen receptor) negative breast cancer patients [5]. Therefore, it is important to identify the mechanism of DACH1 downregulation in breast cancer.

The article "The Function of circRNA-0047604 in Regulating the Tumor Suppressor Gene DACH1 in Breast Cancer" was retracted in 2024. Reasons: signs of a paper mill; suspected computer-generated content; unreliable results or conclusions; concerns about the data.

More and more evidence confirmed that noncoding RNA (ncRNA) plays an important role in mediating breast cancer genesis and progression [6]. MicroRNAs (miRNA) are small noncoding RNAs with nucleotides of 19-25 in length that can regulate posttranscription gene expression. They can combine to the 3′-untranslated regions (UTR) of target mRNAs to block translation [7]. Circular RNAs (circRNAs) belong to the endogenous noncoding RNAs (ncRNAs) which is formed from exons or introns through special selective shearing [8]. It is a single-stranded covalently closed circular transcripts which make it more stable and harder to degrade in cells [9]. Recently, circRNAs have been confirmed as diagnostic biomarkers of many diseases like cardiovascular diseases, rheumatoid arthritis, kidney disease, and cancer [10–13]. Nowadays, the underlying mechanism of circRNA function significantly lies in the miRNA or protein sponges, enhancer of protein function, protein scaffolding, protein recruitment, and templates for peptides translation [9]. So it cannot be overlooked that circRNA plays an important role in regulating tumor-associated genes.

Given that they play a significant role in regulating genes, miRNA is often involved in various biological and pathological processes, such as proliferation, morphogenesis, apoptosis, and carcinogenesis [14]. It is reported that half of human miRNAs are located in cancer-related regions, indicating that miRNA could function as a critical part of tumor development [15]. Accordingly, miRNA is a significant feature in cancer-associated gene dysfunction, and thus, can not only improve cancer diagnosis success rates but also provide a range of clinical applications with targeted research [16]. miR-548o has a highly putative function because it can directly combine to and suppress the expression of DACH1 according to bioinformatics analysis. However, the function of miR-548o in tumor development remains to be researched at length.

Circ_0047604 originated from mothers against decapentaplegic homolog 2 (SMAD2). SMAD family has distinct effects on mammary development and homeostasis [17]. From previous research, upregulate and stabilize SMAD2 protein would contribute to breast cancer progression [18, 19], but the function of circ_0047604 is still unknown.

In this work, we have confirmed that circ_0047604 exerted its antioncogenic role in breast cancer *via* acting as a sponge of miR-548o to regulate DACH1 expression. This study was the first to provide an insight into the mechanism by circRNA regulating DACH1.

## 2. Materials and Methods

### 2.1. Tumor Sample

Tumor and their adjacent normal tissues from breast cancer patients without any treatment before surgery were collected from the Department of Breast and Thyroid Surgery of Shanghai Tenth People's Hospital of Tongji University (Shanghai, China) with patients informed and consent. Our study was approved by Institutional Ethics Committees of Shanghai Tenth People's Hospital (approval number: SHSY-IEC-KY-4.0/17-83/01) and adhered to the standards outlined in the Declaration of Helsinki.

The article "The Function of circRNA-0047604 in Regulating the Tumor Suppressor Gene DACH1 in Breast Cancer" was retracted in 2024. Reasons: signs of a paper mill; suspected computer-generated content; unreliable results or conclusions; concerns about the data.

### 2.2. Cell Culture

The breast cancer cell line MDA-MB-231, MCF-7, and the nonmalignant breast epithelial cell line MCF-10A were acquired from The Chinese Academy of Sciences in Shanghai, China. First, these cells were cultured in a Dulbecco Modified Eagle Medium (DMEM) (Gibco, USA) and supplemented with 10% Fetal Bovine Serum (FBS) (Gibco), penicillin (100 units/ml), and streptomycin (100 *μ*g/ml) (Enpromise, China). Second, these cells were incubated in an incubator at 37°C in a humidified chamber supplemented with a 5% CO_2_ environment. Finally, these cells were split at a ratio of 1 : 3 for every 2-3 days when cell confluence reached approximately 80-90%.

### 2.3. Transfection Assay

The miR-548o mimic, inhibitor, and negative control (NC) were synthesized by Shanghai Genepharma Co., Ltd. (Shanghai, China). Si-RNA specifically targeting hsa_circ_0047606 (si-circ_0047604), negative control (NC) was purchased from IBSBio (Shanghai, China), and a lentivirus plasmid containing circ_0053063 was assembled by ZORIN (Shanghai, China). Plasmid extraction was finished by DNA Midiprep Kits (Qiagen, Hilden, Germany). First, six-well plates were used to culture transfected cells with 1.2 × 10^6^ cells per well. No serum DMEM was added. Second, the MiR-548o mimics, miR-548o inhibitor, circ_0047604 circ_0047604, and (negative control) NC were transfected by using Lipofectamine 3000 (Invitrogen, Carlsbad, CA, USA) according to the manufacturer instructions when the cells reached 30-50%. Third, after 12 hours of incubation, the DMEM medium was substituted for DMEM with 10% FBS. Finally, all cells were incubated at 37°C in a CO_2_ incubator for 36 hours prior to further testing.

### 2.4. Western Blot Analysis

After transfection, cells were washed twice with precooling PBS and resuspended in a RIPA lysis buffer (100 *μ*L/well, Beyotime). After the cell lysate was collected, it was centrifuged for 20 minutes at 4°C (Eppendorf 5804R, Eppendorf Biotech, Germany). The supernatants were collected, and the protein concentrations were quantified using the BCA protein assay kit (Beyotime). 6 × SDS loading buffers (Beyotime) were added to the extracted protein samples, and these samples were degenerated at 100°C for 10 minutes. The total protein was separated by using 10% sodium dodecyl sulfate polyacrylamide gel electrophoresis (SDS-PAGE, Beyotime) and transferred to a 0.45 *μ*m nitrocellulose membrane (Beyotime). This membrane was incubated overnight at 4°C with primary antibodies against DACH1 (1 : 2,000; Bioworld Technology, China) and *β*-actin (1 : 3,000; Bioworld Technology, China). After incubation, the membranes were washed with PBST, and secondary antibodies were used to incubate the washed membranes for 60 minutes at room temperature. Finally, immune reactive protein bands were detected using The Odyssey Scanning System.

The article "The Function of circRNA-0047604 in Regulating the Tumor Suppressor Gene DACH1 in Breast Cancer" was retracted in 2024. Reasons: signs of a paper mill; suspected computer-generated content; unreliable results or conclusions; concerns about the data.

### 2.5. Quantitative Reverse-Transcription PCR (qRT-PCR)

In accordance with manufacturer protocol, the total RNA was extracted from the cells or tissues using TRIzol (Invitrogen, Carlsbad, CA, USA). The PCR parameters for relative quantification were as follows: 2 minutes at 95°C, followed by 40 cycles of 45 seconds at 57°C and 45 seconds at 72°C. The relative expression was evaluated following the relative quantification equation: 2^-*ΔΔ*CT^. Each sample was tested in triplicate. Primers used in this article are presented in Supplementary Table 1.

### 2.6. Dual-Luciferase Reporter Assay

293T cells were seeded in 48 well plates (BD, USA) and cultured until they reached 80% confluence. The mRNA sequence of the hsa_circ_0047604 and DACH1 3′UTR segments, along with the predicted miR-548o binding sites, and the corresponding mutant constructs of the miR-548o binding site was designed and synthesized by IBSBio (Shanghai, China). Cells were cotransected with the constructed reporter plasmids, together with miR-548o or NC using Lipofectamine® 2000 (Invitrogen; Thermo Fisher Scientific, USA). Finally, after 48 hours, firefly and renilla luciferase activities were measured using a Dual Luciferase Assay (Promega, Madison, WI, USA). The firefly luciferase activity was normalized to renilla, and the ratio of firefly to renilla was presented.

### 2.7. Cell Proliferation Assay

The CCK8 assay kit (Sigma, Santa Clara, CA, USA) was applied in accordance with manufacturer instructions to detect for cell proliferation. The transfected cells (2 × 10^3^ cells/well) were seeded into 96-well plates and incubated overnight at 37°C with a 5% CO_2_ environment. Cell proliferation was assessed after replacing medium by 10 *μ*L CCK-8 assays plus 200 *μ*L culture medium per well at 24, 48, 72, and 96-hour intervals. Two hours after incubation, an optical density of 450 nm wavelength was determined at room temperature using a microplate spectrophotometer. Each sample was tested with five replicates.

### 2.8. Wound Healing Assays

Cells were seeded in 12-well plates with 1 mL cell culture medium. After seeding density reach 90%, we produced a scratch by using 1000 *μ*L pipette tip. The scratch area was accessed after 0 h, 24 h by microscope.

The article "The Function of circRNA-0047604 in Regulating the Tumor Suppressor Gene DACH1 in Breast Cancer" was retracted in 2024. Reasons: signs of a paper mill; suspected computer-generated content; unreliable results or conclusions; concerns about the data.

### 2.9. Colony Formation Assay

800 cells were separately seeded in 12-well plates after transfection. After 7 days, when the colonies were visible, the culture was terminated and the plates were washed twice with phosphate-buffered saline (PBS) to remove this medium. These colonies were fixed using 95% ethanol for 10 minutes and dried and stained with 0.1% crystal violet solution for another 10 minutes. Each plate was washed three times with water.

### 2.10. Bioinformation Analysis

A survival analysis of the DACH1 and miR-548o relationship was carried out using patient data by reference to the following website (http://kmplot.com) including all cancer stage and pathological type [20].

The predicted miRNA for targeting DACH1 and miRNA potential target of circRNA was selected by starbase (http://starbase.sysu.edu.cn/) [21]. Expression data including miR-548o and DACH1 relationship was also identified by starbase (http://starbase.sysu.edu.cn/).

### 2.11. Statistical Analysis

This data was calculated using the mean ± the standard deviation (SD) of at least three independent experiments. Student *t*-tests and one-way ANOVA were used to evaluate the differences between each group using SPSS 20.0 software. These differences were considered significant for *P* values < 0.05.

## 3. Results

### 3.1. Breast Cancer with Low Expression of DACH1 Has a Poor Outcome in Breast Cancer Patients, and DACH1 Is Underexpressed in Breast Cancer Cell Line

A lower level of expression was found for DACH1, and this has been related to tumor development and progression [22–24]. The DACH1 expression level in 1809 patients was analyzed using Kaplan-Meier Plots. It was shown that this lower level of expression in breast cancer was significantly correlated with a lower survival rate as showed in Figure 1(a). The expression level of DACH1 in the MDA-MB-231, MCF-7, and MCF-10A breast cancer cell lines was further identified. These results show that the DACH1 expression level is also downregulated and is consistent with reported clinical results (Figure 1(b)).

### 3.2. miR-548o Directly Targets DACH1 in Breast Cancer Cells

The database of starbase indicated a strong possibility that miR-548o could be a candidate regulator in binding microRNAs to DACH1 mRNA (Figure 2(a)). To investigate whether miR-548o can bind to DACH1 3′-UTR, a luciferase reporter assay was carried out in 293T cells. The DACH1 original 3′-UTR predicted region was replaced by a mutation sequence as shown in Figure 2(b). As shown in Figure 2(b), the luciferase activity decreased after cotransfection with psi-CHECK-2/DACH1 3′-UTR and miR-mimics in comparison with control groups. This supports that miR-548o specifically binds to the 3′-UTR of DACH1 mRNA. From correlation between miRNA-548o and DACH1 expression level, it is shown that miRNA-548o and DACH1 showed negative correlation in 1085 breast cancer samples (Figure 2(c)). miR-548o showed a higher expression level, and higher expression of miR-548o showed a poorer survival rate (Figures 2(d) and 2(e)).

The article "The Function of circRNA-0047604 in Regulating the Tumor Suppressor Gene DACH1 in Breast Cancer" was retracted in 2024. Reasons: signs of a paper mill; suspected computer-generated content; unreliable results or conclusions; concerns about the data.

### 3.3. Increase miR-548o Expression Level Will Promote the Proliferation of Breast Cancer Cells

Given that miR-548o has an absent function in tumors, the miR-548o mimics and the miR-548o inhibitor were transfected into MDA-MB-231 and MCF-7 cells to investigate the impacts of miR-548o functions in breast cancer cells. CCK8 assays were used to assess cell proliferation at 24, 48, 72, and 96-hour intervals after the miR-548o mimics and inhibitor were transfected and proliferation abilities was calculated. As shown in Figure 3(a), miR-548o mimics can promote cell proliferation in a time-dependent manner, while the miR-548o inhibitor produced opposite results. The colony formation assays (Figure 3(b)) also showed the same trend because miR-548o formed colony areas were more and larger than those formed under negative controls, while the miR-548o inhibitor produced opposite results. Ultimately, these results revealed that an overexpression of miR-548o can promote a cellular proliferation ability.

Further research into the migration role of miR-548o in mediating breast cancer was identified using wound healing assay. Cells transfected with miR-548o mimics and miR-548o inhibitor groups were compared to miR-NC and miR-NC inhibitor transfection groups. As is shown in Figure 3(c), the miR-548o mimics group showed an apparently smaller scratched area, while the miR-548o inhibitor group showed a contrary trend.

### 3.4. Circ_0047604 Is an Important Factor to Regulate miR-548o

Recent research revealed important treatment with wild-type circ_0047604 showed decreased luciferase activity, but not the mutation-type (Figure 4(b)). From western blot assays, it shows that increased circ_0047604 would upregulate DACH1 level and decreased circ_0047604 would inhibit DACH1 expression (Figure 4(c)). We further tested the DACH1 and circ_0047604 expression level. As Figures 4(d) and 4(e) show, both DACH1 and circ_0047604 expressed significant lower in tumor tissues than that in normal tissues. Pearson correlation analysis of DACH1 expression and circ_0047604 expression in 11 samples showed a markedly positive correlationship (Figure 4(f)).

### 3.5. Circ_0047604 Can Inhibit Cancer Cell Proliferation and Migration

At last, we further test the function of circ_0047604. Circ_0047604 can inhibit breast cancer cell proliferation (Figure 5(a)). The colony formation assays (Figure 5(b)) also showed the same trend. From wound healing assays, it is shown that overexpressed circ_0047604 can inhibit cell migration and inhibition of circ_0047604 could act as a carcinogenic factor.

The article "The Function of circRNA-0047604 in Regulating the Tumor Suppressor Gene DACH1 in Breast Cancer" was retracted in 2024. Reasons: signs of a paper mill; suspected computer-generated content; unreliable results or conclusions; concerns about the data.

## 4. Discussion

According to recent studies, DACH1 is identified as an important marker related to breast cancer prognosis [25]. These studies indicate that the presence of DACH1 in different tumors indicates that it can suppress the growth and invasion of tumor cells through a signal pathway in a variety of researches [26–29]. Previous reports have implicated that DACH1 could suppress tumor cell proliferation, migration, and invasion by mediating other important biomarkers, such as Estrogen Receptor-*α*, Peroxiredoxin 3, Wnt/*β*-catenin signaling Smad4, and TGF-*β* [5, 30–33].

MicroRNA is often involved in many aspects of biology, including embryogenesis, aging, metabolism, and immunity. However, the microRNAs related to the pathogenesis and progression of various human diseases are considerably more important [34]. A novel class of drugs called anti-mirs and miRNA-mimics capable of regulating miRNA level is currently in various stages of preclinical and clinical testing. This brings about the hope that someday a miRNA-based therapeutic approach can be used to treat common human diseases [35]. The function of miR-548o on tumors has not yet been reported, and almost no research has been conducted on miR-548o. In this study, it has been shown that miR-548o can regulate DACH1 expression directly and can enhance both the proliferation and migration of breast cancer cells *in vitro*. Normally, microRNAs could be grouped in relation to their function into two types: onco-miRs (an oncogene-like microRNA) or tumor suppressor-miRs (a tumor suppressor-like microRNA) [36]. Preliminary results showed that miR-548o could be regarded as an oncogene-like microRNA by regulating DACH1 expression, and miR-548o could be regarded as a tumor oncogene-like miRNA involved in mediating breast cancer.

Recent reports indicate that circRNA can act as miRNA sponge and interacting with proteins to affect gene expression level to influence transcription and translation [37–39]. After further analyzing circRNA on breast cancer sample, we found that circ_0047604 expression level is lower in tumors. It could bind to miR-548o and, to a large degree, also affect DACH1 expression. Considering that circ_0047604 is originated from SMAD2 gene and SMAD2 always acts as an oncogenic gene in breast cancer [40], it means circ_0047604 exerts contrary to original SMAD2 protein. Therefore, the relationship between SMAD2 mRNA transcription and circRNA production is not clear and still needs further investigation. More clinical cases, different tumor progressions, and other physiological processes are needed.

The article "The Function of circRNA-0047604 in Regulating the Tumor Suppressor Gene DACH1 in Breast Cancer" was retracted in 2024. Reasons: signs of a paper mill; suspected computer-generated content; unreliable results or conclusions; concerns about the data.

## Figures and Tables

**Figure 1:** Survival related to expression level of DACH1 and its expression level in cell lines. (a) The expression level of DACH1 relationship with survival rate. (b) The expression level of DACH1 is also lower in MCF-7 and MDA-MB-231 compared with MCF-10. The graph represents the compared values ± SD; ^∗∗∗^*P* < 0.001.

**Figure 2:** DACH1 is a direct target of miR-548o. (a) The binding site for miR-548o in 3′-UTR of DACH1 mRNA. (b) The coexpression level between DACH1 and miR-548o. (c) The wild and the mutation sequence of the binding site. The relative luciferase activity was measured in 293T cells after cotransfecting the DACH1 luciferase construct with either miR-548o or NC. (d) The expression level of miR-548o. (e) The expression level of miR-548o relationship with survival rate. ^∗^*P* < 0.05, ^∗∗^*P* < 0.01, ^∗∗∗^*P* < 0.001.

**Figure 3:** miR-548o can promote tumor cell growth and immigration. (a) The CCK-8 assay was carried out to monitor the proliferation level of MDA-MB-231 and MCF-7 cells at 1, 2, 3, and 4 days. (b) Images of crystal violet stained colonies of MDA-MB-231 and MCF-7 cells transfected with NC, miR-548o, and miR-548o inhibitor. (c) Wound healing assays to test cell migration after transfection of NC, miR-548o, and miR-548o inhibitor. ^∗^*P* < 0.05, ^∗∗^*P* < 0.01, ^∗∗∗^*P* < 0.001.

**Figure 4:** Circ_0047604 can be a sponge of miR-548o. (a) The binding site for miR-548o in circ_0047604. (b) The wild and the mutation sequence of the binding site. The relative luciferase activity was measured in 293T cells after cotransfecting the circ-0047604 luciferase construct with either miR-548o or NC. (c) DACH1 expression level after up/downregulating circ_0047604. (d) and (e) The expression levels of DACH1 and circ_0047604 in tumor tissues. (f) The coexpression level between DACH1 and circ_0047604. ^∗^*P* < 0.05, ^∗∗^*P* < 0.01, ^∗∗∗^*P* < 0.001.

**Figure 5:** Circ_0047604 can inhibit tumor cell growth and immigration. (a) The CCK-8 assay was carried out to monitor the proliferation level of MDA-MB-231 and MCF-7 cells at 1, 2, 3, and 4 days. (b) Images of crystal violet stained colonies of MDA-MB-231 and MCF-7 cells after up or downregulation of circ_0047604. (c) Wound healing assays of cell migration after up or downregulation of circ_0047604. ^∗^*P* < 0.05, ^∗∗^*P* < 0.01, and ^∗∗∗^*P* < 0.001.

The article "The Function of circRNA-0047604 in Regulating the Tumor Suppressor Gene DACH1 in Breast Cancer" was retracted in 2024. Reasons: signs of a paper mill; suspected computer-generated content; unreliable results or conclusions; concerns about the data.

## Data Availability

All data included in this study are available upon request by contact with the corresponding author. Pro. Lin Fang, Department of Breast and Thyroid Surgery, Shanghai Tenth People's Hospital, Tongji University, 301 Yanchang Road, Jing'an Area, Shanghai 200072, China. E-mail: fanglin2017@126.com; Pro. Yuanzhi Xu, Department of Stomatology, Shanghai Tenth People's Hospital, Tongji University School of Medicine, 301 Yanchang Road, Shanghai 200072, China. E-mail: amyxyz01@hotmail.com. Dr. Bingkun Zhao, Department of Breast and Thyroid Surgery, Shanghai Tenth People's Hospital, Tongji University, 301 Yanchang Road, Jing'an Area, Shanghai 200072, China. E-mail: zhaobingkun0506@163.com.

## Supplementary Materials

Supplementary Materials Supplementary Table 1: nucleotide sequences of primers used for qRT-PCR.
